# Detection of Breast Cancer from Five-View Thermal Images Using Convolutional Neural Networks

**DOI:** 10.1155/2022/4295221

**Published:** 2022-02-28

**Authors:** Mathew Jose Mammoottil, Lloyd J. Kulangara, Anna Susan Cherian, Prabu Mohandas, Khairunnisa Hasikin, Mufti Mahmud

**Affiliations:** ^1^Intelligent Computing Lab, Department of Computer Science and Engineering, National Institute of Technology, Calicut, PO Box: 673601, Kerala, India; ^2^Department of Biomedical Engineering, Faculty of Engineering, Universiti Malaya, Lembah Pantai 50603, Kuala Lumpur, Malaysia; ^3^Center of Image and Signal Processing (CISIP), Faculty of Engineering, Universiti Malaya, Lembah Pantai 50603, Kuala Lumpur, Malaysia; ^4^Department of Computer Science, Nottingham Trent University, Clifton Lane, Nottingham, NG11 8NS, UK

## Abstract

Breast cancer is one of the most common forms of cancer. Its aggressive nature coupled with high mortality rates makes this cancer life-threatening; hence early detection gives the patient a greater chance of survival. Currently, the preferred diagnosis method is mammography. However, mammography is expensive and exposes the patient to radiation. A cost-effective and less invasive method known as thermography is gaining popularity. Bearing this in mind, the work aims to initially create machine learning models based on convolutional neural networks using multiple thermal views of the breast to detect breast cancer using the Visual DMR dataset. The performances of these models are then verified with the clinical data. Findings indicate that the addition of clinical data decisions to the model helped increase its performance. After building and testing two models with different architectures, the model used the same architecture for all three views performed best. It performed with an accuracy of 85.4%, which increased to 93.8% after the clinical data decision was added. After the addition of clinical data decisions, the model was able to classify more patients correctly with a specificity of 96.7% and sensitivity of 88.9% when considering sick patients as the positive class. Currently, thermography is among the lesser-known diagnosis methods with only one public dataset. We hope our work will divert more attention to this area.

## 1. Introduction

Cancer is among one of the most predominant diseases prevalent today. Among its various types, breast cancer has become quite notable. Breast cancer can affect both males and females. It affects more than 2.3 million women, which accounts for more than 11% of the total cancer cases in the world as stated by GLOBOCAN 2020 [1]. Meanwhile, cases in men are rare, having an incidence rate of 0.5–1% [2].

Breast cancer accounts for 14% of cancers in India. Kerala records the highest cancer rates as compared to the rest of the country. When considering breast cancer specifically in Kerala, it is quite common among women, accounting for 30–35% of the cancer cases. A prevalence rate of 19.8 per 100,000 and 30.5 per 100,000 was observed in rural and urban areas, respectively, as per the Thiruvananthapuram Cancer Registry [3]. This could be attributed to the increasing elderly population in Kerala, accounting for nearly 20.9% of their population by 2031.

Studies have shown an increment in the occurrence of breast cancer among the younger population as opposed to 25 years ago in India. About 25 years ago, 69% of the affected individuals were above 50. However, trends show that approximately 48% of them are below the age of 50. Breast cancer was found to account for 23–32% of the cancer cases in women by 2012, overtaking cervical cancer as the most prevalent cancer type [4].

Older women (age greater than 65) have a greater chance of having breast cancer when compared with younger women (age less than 35). Hence, many young women do not undergo cancer detection screenings until the age of 40. Due to this, the survival rates among the younger affected population are much lower than what is observed for affected women of ages 65–74. [5]

There are several treatments available today that try to combat the effects of breast cancer. These include surgery to remove cancerous cells, chemotherapy, and radiation. With rising cases and increasing mortality rates, breast cancer has become a major medical concern within society.

A convolutional neural network is built, which considers five thermal views of the breast along with the patient's clinical data. This then is used for the classification of the patient as healthy or sick. The main contributions of this work include the following:

- Performance comparison of single-input CNN and multi-input CNN to see which one gives better predictions
- Providing experimental proof to show that adding clinical data improves the prediction of the model
- Coupling results of a thermography with the other screening techniques can help improve prediction results

In this paper, the section organization is as follows.  Section 2 takes a closer look at the origin of the problem and the problem statement that is being worked on. An extensive review of breast cancer and the existing work done for its identification is discussed in Section 3. Details regarding the dataset and the data collected are outlined in Section 4. Sections 5 and 6 present the methods for creation of model and data preparation. Results are discussed in Section 7. Conclusion and future plans are mentioned in Section 8.

## 2. Problem Statement

### 2.1. Origin of Work

Breast cancer is a prevalent form of cancer in women. Over the years, there has been significant amount of research that incorporates machine learning principles to help predict the existence of cancerous cells in the breast with high accuracy. Further studies have been done in the localization of such regions which helps radiologists study it further and provide the necessary treatments. In [6], the authors have tried machine learning algorithms to predict the presence of cancer using thermal images of the breast. The most common screening technique currently used is mammography which has disadvantages such as exposure to radiation, high costs to get a screening, and discomfort to the patient. Paper [6] is among the first few papers that worked on adding clinical data of the patient to the multi-input convolutional neural network.

### 2.2. Problem Definition

Detection of breast cancer is a challenging task and can be life-threatening if not detected at an early stage. There are many tools and technological advances to detect breast cancer. Mammography has become a popular screening technique. However, mammography exposes the patient to radiation and causes discomfort to the patient. Thermographic screenings require no contact with the machine and are lower in cost than mammography enabling patients to get screenings more often. The advancement of artificial intelligence technology has enabled a deep neural network approach in aiding medical practitioners in rapid diagnosis [7, 8]. The convolutional neural network designed uses multiple thermal views of the breast for each patient from the benchmark dataset. It compares the effect of the addition of clinical information collected of each patient to the model.

## 3. Literature Review

Breast cancer can be detected using many methods; some of them are discussed in Table 1. Thermography is considered a less invasive and cost-efficient screening technique compared with mammograms [16]. Mammography requires the patient to have contact with some machinery during the process, but thermography requires no contact while screening. Furthermore, there is no exposure to radiation that would otherwise arise if mammography was done. Thermography could also be used to diagnose women of all ages with any breast density, hence, making thermography more suitable.

Due to the aggressive nature of breast cancer and its rapid multiplicity, the cells will expend a lot of energy because of the repeated cell divisions. Hence, the presence of lesions on the breast can be detected due to this temperature difference. For this study, images were collected using quantitative thermography. The main reason is because the presence of tiny lesions for the early detection of cancer is significant and such temperature differences should be collected for each pixel to get a complete in-depth view of the patient's breasts. When qualitative thermography is used, an in-depth detailed image of the breast is not obtained, and such images may not be able to correctly differentiate the slight temperature variations which detect the early presence of cancer. A quantitative measurement camera can also provide the temperature variations of such regions with the rest of the body which can help any model in detecting the presence of cancer.

Table 2 shows the different approaches of detecting breast cancer using thermal images. The popularity of thermography is relatively quite recent. Earlier thermal images were analyzed by humans making the process strenuous and inaccurate. With the emergence of artificial intelligence (AI) and machine learning (ML) algorithms, thermal images can be intercepted and used in a whole new different way. Thus, it makes thermography a very powerful method that can overcome the disadvantages of mammograms [28, 29].

Currently, there are not many studies that test the efficiency of thermograms in predicting the possibility of breast cancer. Hence, devising a model along these lines could contribute to the ongoing research in this area.

### 3.1. Observations

Breast cancer has risen to be one of the most widespread cancer types with a significant fatality rate depending on various factors such as age. Early detection is a crucial method to combat this disease. Compared to relatively older women (above 65 years old), adolescents and teenagers have a much lower probability of being diagnosed with breast cancer. This is mostly because breast cancer screening is done after they are 40. Three methods discussed in this report for early detection include mammography, clinical, and self-examination. The convolution neural network implementation has been made to predict breast cancer.

The CNN mechanism classifies the image by breaking it down into its features, reconstructing it, and predicting it at the end. The edge-based samples have been considered to reduce the comparison time and space. This results in increased accuracy. The reason for picking thermography over mammography is, as mentioned in the report, the boom of AI opened new possibilities, and thermography being a contact-less screening method makes it more preferred over mammography. The idea behind adding clinical data along with the thermal images is that it enhances the accuracy of the model, as exhibited in [6].  Table 3 shows some pros and cons regarding certain other approaches discussed earlier.

### 3.2. Impact of Technology on Breast Cancer Prediction

Technology has a lot of impact on the early prediction of breast cancer. Image processing is a very important component for its prediction. Some of the techniques used to obtain images are computerized tomography (CT) scan, MRI, mammograms, thermography, and ultrasound. One very important application of using technology is that they can be used to identify and detect regions of growth and segment those regions and radiologists can use this to study cancers and help the patients [34].

#### 3.2.1. Artificial Neural Network

One of the most important uses of artificial neural networks is their ability to be used in place of mammography and breast MRIs where they can be used to screen severe cases of cancer. ANNs can be used to detect cancer and can be used to find benign tumours as efficiently and accurately as possible [35]. Mammography can be expensive and as the patient is exposed to radiation, mammography cannot be used as a screening tool at regular intervals. Mammography can cause patients some discomfort which is eliminated when using neural networks in the early detection of breast cancer.

#### 3.2.2. Convolutional Neural Network

Convolutional neural networks have the ability to extract complex features from any image that it processes [36]. They help us find patterns that are common among different images. The basic operation which is performed here is that, for each cell or pixel in the image matrix, the cell is multiplied by an element in the weight matrix, followed by the addition of the resulting products. Going through a CNN, the first few layers can help us identify edges in the image, and going deeper in the network, extracts more information from them. Moving across the network, we reduce the dimensions of an image, while retaining the important information used to make a prediction.  Table 4 shows some CNN models prevalent today.

## 4. Materials

### 4.1. Mammographic Images Dataset

#### 4.1.1. Digital Mammography Dataset

This dataset consists of only the clinical data generated from around 40,000 mammograms (20,000 digital mammograms and 20,000 film screen mammograms) collected between the years 2005 and 2008 by the Breast Cancer Surveillance Consortium. The clinical data includes mammogram assessment, details on breast cancer diagnosis within one year, age of the patient, family history of breast cancer, biopsy details, breast density, etc. [40].

#### 4.1.2. MIAS Mini Mammography Database (i.e., Mini-MIAS Database of Mammograms)

Dataset consists of digital mammograms which were collected by the Mammographic Image Analysis Society. The dataset consists of 322 images from 161 patients containing the right and left views of the breast for a single patient. Each image has a resolution of 50 microns. Details of the presence of any abnormalities are also mentioned in the dataset. All the images in the dataset are in grayscale format with a size of 1024 × 1024 pixels. This dataset was compiled in 2015 and its version is 1.21 [40, 41].

#### 4.1.3. Digital Database for Screening Mammography (DDSM)

The dataset of mammograms consists of 2500 studies where each sample consists of two images of the breast along with the patient's clinical information such as breast density; presence of abnormalities is also mentioned in the dataset. The resolution of the images ranged from 42 microns to 50 microns. The images collected were classified as either normal, benign, or malignant. The datasets were compiled by Massachusetts General Hospital, Sandia National Laboratories, and the University of South Florida Computer Science and Engineering Department [42].

### 4.2. Thermographic Images Dataset

Thermography is a detection method that uses an infrared camera to identify heat patterns based on the infrared emissions given off by an individual. Database for Mastology Research (DMR) [43] is an online platform that stores and manages mastologic images for early detection of breast cancer. This database includes the data of the patients from University Hospital Antonio Pedro (HUAP) of the Federal Fluminense University of Brazil.

The database contains data from 293 patients. The database includes thermal images (front, lateral views), thermal matrix (where each pixel contains the thermal information), and clinical and personal information (this includes menstrual details, medical history, data acquired as part of protocols, previously diagnosed positive or negative, age, and eating habits) of the patient. There are two protocols that are used in thermography because the whole point of the thermogram is to note how the body cells react under different temperature conditions.

Static protocol: patients will be asked to rest themselves with the help of brackets, whilst frontal and lateral views (including right, left, right oblique, and left oblique views) imagery will be captured. The whole point of this is for the patient to attain thermal stability.

Dynamic protocol: once the thermal stability is acquired, the patient will be subjected to cooling using a conditioning fan. Frontal and lateral images are obtained sequentially (5-second gap).

Images are recorded using a FLIR SC620 thermal camera which is captured using the static and dynamic protocols. Their dimensions were 640 × 480.

## 5. Methods

### 5.1. Steps for Predicting Breast Cancer Using Thermal Images

The dataset was obtained from the Database for Mastology Research (DMR). The thermal images of five different views (front, left 45°, right 45°, left 90°, and right 90°) of the breasts were used. Along with this, the clinical data of each patient was recorded using web scraping.

After the extraction of thermal images and clinical data, we moved on to image and data preprocessing. The images that we collected were of dimensions 640 × 480. Patients that had fuzzy images, images that did not follow protocol, or did not have all five views were removed from the dataset. For data preprocessing, any anomalous entries were deleted as well. In the current implementation, the CNN models that were built and trained worked for square images. Hence, as part of data preprocessing, all the images were transformed to images of size 640 × 640. To transform each image to a square image, the resize functionality provided by PyTorch was used. After this, it passes through various classification methods as shown in Figure 1.

### 5.2. Architecture Diagram

Once the image and clinical data preprocessing is completed, the focus shifts to building models that could be used for classification. In the current design, a convolutional neural network is built for each of the five views of the breast. Each model is trained separately to make sure that they perform well individually before combining their output. The output of each model will be a tuple containing the probability of the patient being sick and the probability of the patient being healthy. The probability of a patient being diagnosed as healthy is denoted by P(H) and the likelihood of a patient being diagnosed as sick is P(S).  Table 5 shows the output that would be generated by each model.

Once the training of the five neural networks is completed, the results will be combined to train the final neural network. The combined result will be a 10-element tuple such that each of the 5 views will contribute the probability of a healthy and sick diagnosis. The set of these tuples for all of the patients who were part of the training data is then used to build and train the final neural network. The resulting output of the final neural network will be the prediction of healthy or sick by the multi-input CNN model.

The next step is to add personal and clinical data to the model and see the change in the performance of the model after appending the result of the model that was trained on the clinical data. The clinical data collected includes information about the age, conditions, symptoms, family history, menarche, etc. Once categorization of this dataset is completed, a neural network is built for the clinical data. The output of this neural network will be a value between 0 and 1. A threshold of 0.5 is set to decide if the prediction is healthy or sick.

- If P (clinical data) < 0.5, patient diagnosis prediction: healthy
- If P (clinical data) > 0.5, patient diagnosis prediction: sick

Once this clinical data neural network model is trained, its output will be appended to the output of the multi-image CNN model giving an 11-element tuple which would be passed as input to the final neural network. Both images and clinical data are treated separately and only the outputs from their respective models (i.e., CNN for images and neural network for clinical data) are concatenate to determine the final classification. Different performance evaluation metrics are run on the final neural network to see how the addition of clinical data to the model affects its performance. A detailed overview of the steps followed to obtain the prediction using thermal images alone and thermal images along with clinical data is shown in Figure 2.

## 6. Data Preparation

The images are recorded using a FLIR SC620 thermal camera, which is captured using static and dynamic protocols (to see details of each protocol, refer to the dataset section of the report). The different views captured are shown in Figure 3.

### 6.1. Image Preprocessing

(i) Identify the inaccurate or incomplete entries, then either try to rectify it or delete the entry. The same is applied to thermal and personal clinical data
(ii) All patients that did not have all five views (i.e., front, left 45°, right 45°, left 90°, and right 90°) were removed from the dataset
(iii) If the static view of a front or lateral view was not available or was fuzzy, we replaced them with images taken with the dynamic protocol
(iv) Images will be removed if they are as follows:
  - Blurry and barely visible (refer to Figure 4(a))
  - Presence of injury (refer to Figure 4(b))
  - Proper protocols were not followed during the process of data collection (for example, keeping arms down or images taken from a different angle) (refer to Figure 4(c))

### 6.2. Clinical Data Preprocessing

(i) Since the database was procured from Brazil, the text had to be converted to English
(ii) Patient's age was constantly updated in the database which was converted to the age at the time of visit
(iii) Some cases such as Patient 398 had their age as 0 and Patient 211 had their age as 120. Such anomalies were removed
(iv) All entries which were blank were filled appropriately with values such as “not answered”
(v) (Patient's age was constantly updated in the database which was converted to the age at the time of visit
(vi) Some cases such as Patient 398 had their age as 0 and Patient 211 had their age as 120. Such anomalies were removed
(vii) All blank entries were filled appropriately with values such as “not answered”
(viii) The final set of features included the following:
  - Discrete features: diagnosis, marital status, race, complaints, symptoms, signs, menopause, eating habits, family history, cancer family, mammography, radiotherapy, plastic surgery, prosthesis, biopsy, use of hormone replacement, signs of wart on breast, smoking habit, drinks coffee, consumes alcohol, physical exercise, applied products, visible nipple changes and body temperature
  - Continuous features: age at time of screening and menarche age

### 6.3. Construction of Classification Model

There are three kinds of CNN layers:

- Pooling layer
- Convolutional layer
- Fully connected layer

Using these layers, each thermal image is gone through the models independently and their output is concatenated to predict the outcome of the disease.

### 6.4. Performance Evaluation Metrics

#### 6.4.1. Current Dataset after Preprocessing

After preprocessing, there are 157 healthy patients and 84 sick patients. This is split into 80% for training set and 20% for test set as shown in Table 6. The 80/20 ratio is the most common combination of splitting training set and test set which can provide the best results. In general, 70–80% is used for training and the remaining 20–30% for testing.

#### 6.4.2. Formulas Used for Model Evaluation

The sick class is considered positive, while the healthy class is deemed to be negative.  Table 7 outlines the metrics used for the evaluation of the models.

## 7. Results and Discussion

### 7.1. Loss, Optimizers, and Normalizing Functions

For all the models discussed below, a Stochastic Gradient Descent (SGD) optimizer was used. The Adam optimizer was also tried; however, it was noticed that the model was overfitting very quickly and it was negatively affecting the overall diagnosis prediction. When SGD was used with a learning rate of 0.001, the loss reduced after each epoch, and training of the model was stopped after a certain number of epochs before the loss started to flatten. To calculate the loss between the actual value and predicted value, Cross Entropy Loss function was used.

Before the data was passed through the ANN, the data was normalized. This was done using the MinMaxScaler. The reason the scalar is used is to remove any form of bias before passing it to an ANN so that the decision-making process of the neural network may not be affected by any other external factor. The models were trained batch-wise so that the models could see different sets of inputs to improve its performance.

### 7.2. Model 1: Same Architecture for All 3 Views

In the current implementation, the models use 3 views of the thermographic images of the breast (frontal, left 90°, and right 90°). The model in Figure 5 uses convolutional layers with channel sizes of 32, 64, and 128. We use strides with a value of 2 and pooling layers of size 2 × 2 to reduce the matrix size from 640 × 640 × 1 to a 1 × 2 matrix containing the probabilities. In this multi-input CNN, the same convolution neural network architecture was used to train all three views and their outputs were combined. After this, another model that combines the result of the three CNNs and the neural network trained on the clinical data is built. The results of the model were evaluated with the same model after the decision from the clinical data was added.

#### 7.2.1. Model Performance

Model 1 had an accuracy of 85.4% without clinical data and 93.8% with clinical data. The proportion of sick patients that got classified correctly is about 77.8% without clinical data and it increased to 88.9% after the addition of clinical data decision. Similarly, 90% of the healthy patients got classified correctly without clinical data and was 96.7% after the addition of clinical data decision. The performance scores of the model are mentioned in Table 8.

The area under the ROC curve is around 0.89 without clinical data and 0.987 with clinical data. As this dataset has a class imbalance and since we are more interested in the prediction of sick patients, we calculate the precision and recall and the curve associated with them. We see that a perfect predictive model would have a curve at (1,1). The precision-recall curve is seen to be tending towards (1,1) indicating that the model is performing well. The AUC score for this precision-recall curve is 0.841 without clinical data and 0.977 with clinical data. The plots for the model with and without clinical can be seen in Figure 6.

To give a better perspective, a blue dotted line is drawn on both graphs to denote a model that has no skill; i.e., it simply outputs a prediction randomly. If the graph of the model, here, the multi-input CNN, is above this line (as is seen by the ROC curve and the precision-recall curve), it signifies a much better performance than the no skill model.

### 7.3. Model 2: Different Architectures for Frontal and 90° Views

This model also uses the 3 views of the thermographic images of the breast (frontal, left 90°, and right 90°). In the model in Figure 7, the left and right views use the same CNN model with channels of size 45, 90, 135, and 180 while the front view uses a different model with channels of size 50, 100, 150, and 200. The multi-input CNN reduces the image to output probabilities of size 1 × 2. The results of the model along with its performance in comparison with clinical data are also mentioned in Table 9.

#### 7.3.1. Model Performance

Model 2 had an accuracy of 81.2% without clinical data and 89.6% with clinical data. The proportion of sick patients that got classified correctly is about 75.0% without clinical data and 87.5% after the addition of clinical data decision. Similarly, 84.4% of the healthy patients got classified correctly without clinical data and it increased to 90.6% after the addition of clinical data decision. The area under the ROC curve is around 0.802 without clinical data and 0.900 with the addition of clinical data decision. The AUC score for this precision-recall curve is 0.771 without clinical data and increases to 0.923 after the addition of clinical data decision. The plots for the model with and without clinical can be seen in Figure 8.

### 7.4. Discussion

#### 7.4.1. Clinical Data

Symptoms such as irritation and rashes are common in women with breast cancer. Research also shows that factors such as age [44] or hormone replacement [45] play a role in the disease. Such data coupled with the thermal images would add value as they give a more extensive idea of the patient and their health.

The models created so far have been able to perform with high accuracy after adding the patient's clinical information as seen from their performance. There are some signs and symptoms that can indicate cancerous cells in the body. Hence, such clinical information can effectively predict the presence of breast cancer. After collecting the patient's information, it is passed through an ANN. ANNs use backpropagation that helps to identify which features are more important and then use this information to make a decision.

Since the features collected are general to any patient, this information can be used for any other problem. For example, if any other cancer such as lung cancer was being detected, the same ANN can be used to train the model with the patient's diagnosis. The ANN then learns which feature is most important for the problem of lung cancer and uses that information to make a decision. Hence, the addition of clinical data is a very easy and effective tool to diagnose a patient, and thus it can be used for a variety of purposes.

Currently, it was observed that most datasets only collect the images of the different screening of a patient and use it to make a decision. This work aims to encourage more people to start collecting clinical data along with the images and use this information also to make a diagnosis prediction.

#### 7.4.2. CNN

Generally, the CNN used to classify the frontal images was able to classify both the healthy and sick patients with an accuracy above 0.7. When different CNN models were being trained for the different views, it was noticed that the models were able to classify either healthy samples or sick samples with high accuracy while the other class had an accuracy of 0.6. In such cases, different epochs for the different models were tried and the final model was built after ensuring that they perform their best individually. The performance of the models that handle each view before the combination of their results is shown in Table 10.

Data augmentation techniques are mainly used when the dataset is small to generate more samples for the model to learn better. Multi-view CNNs perform better than single-view CNN. In multi-view CNN, different views of the same object are being used as input, so information and features generated from each image can be pooled together to improve the prediction. And data augmentation techniques have been used to complement or improve the performance of the multi-view CNNs [46].

Quantitative comparison of our work with other methods using thermographic images is shown in Table 11.

## 8. Conclusion

From the current work, it is found that the addition of clinical data to the convolutional neural networks increased the ability of the model to classify a patient as healthy or sick correctly. We see an accuracy of 93.8% for the model that uses data over 85.4% for the one that does not. Addition of clinical data helps in strengthening the prediction of breast cancer using CNN models. These findings could also bring to light the importance of increasing the research in the area of thermography. Increased research could improve the techniques employed for thermography and thus help it to become a standard in breast cancer detection in the future.

Since only a multi-input CNN was used for classification, a comparative study of the performance of a single-input CNN with the current input is planned. Along with this, another possible experimental study is using pretrained CNN models for classification. Some techniques for data preprocessing that could be explored are data augmentation and image segmentation. It is interesting to see how each model interacts with the limited data available.

## Figures and Tables

**Figure 1:** Different methods employed for prediction.

**Figure 2:** Design of the multi-input CNN.

**Figure 3:** The views: (a) Front. (b) Left 45°. (c) Left 90°. (d) Right 90°. (e) Right 45°.

**Figure 4:** (a) Fuzzy frontal view. (b) Protocol not followed. (c) Injury on the breast. (d) Clear frontal view.

**Figure 5:** Multi-input CNN model 1. (a) CNN model for front view, (b) CNN model for right 90° view, (c) CNN model for left 90° view.

**Figure 6:** Model 1 AUC plots. (a) ROC curve without CD, (b) precision-recall curve without CD, (c) ROC curve with CD, (d) precision-recall curve with CD.

**Figure 7:** Multi-input CNN model 2. (a) CNN model for front view, (b) CNN model for right 90° view, (c) CNN model for left 90° view.

**Figure 8:** Model 2 AUC plots. (a) ROC curve without CD, (b) precision-recall curve without CD, (c) ROC curve with CD, (d) precision-recall curve with CD.

**Table 1:** Machine identification methods.

Methods	Description
CT scan	It provides x-ray images that give a complete cross-sectional view of the internal organs. It has a significant advantage in evaluating of the breast to identify cancerous cells. CT scans are used for more advanced stages of cancer to check if cancer has spread to other parts of the body or to see the effects of medication on the cancerous cells [9].
MRI scan	It uses radio waves to produce scans of the body. It is used to determine the presence of cancerous cells in the body and to see the tumor's growth region. It does not expose a person to radiation, hence a safer alternative to mammograms. In certain cases, a gadolinium-based dye or contrast material could be injected into the arm to show the images more clearly [10].
Mammograms	It produces an x-ray of the breast used for early detection of breast cancer. During this procedure, the breasts are compressed by compression plates. It is one of the most effective methods for detecting breast cancer when no lump is visible or when the patient would like to scan any specific area that shows certain symptoms associated with the disease. If a woman has a high risk of breast cancer, screening starts at a younger age [11, 12].
Ultrasound	It uses sound waves to produce images of the breast. It is not usually employed as a screening tool, but is used along with a mammogram to find the existence of a fluid filled cyst or tumour. They are similar to thermography where there is no exposure to radiation and are effective for women with dense breasts, pregnant women, and young women (age below 25) [13].
Thermography	It captures the image of breasts using a device which essentially evaluates the surface temperature of the skin of the breasts. During this screening process, there is no radiation, no contact between the patient and the device, and no breast compression, making it a desirable screening tool. It is based on the principle that we know cancer cells grow and spread to different regions fast due to their high metabolism. As metabolism increases, the temperature at that region also increases which can be used to detect the presence of cancerous cells [14, 15].

**Table 2:** Papers outlining different approaches to breast cancer detection using thermal images.

References	ML approach	Dataset used	Classification	Evaluation metrics
Schaefer et al. [17]	If-then rules	146 images (29-malignant 117-benign)	Fuzzy rule-based classification	Classification 78.05%, sensitivity 74.14%, specificity 79.02%
Abdel-Nasser et al. [18]	Learning to rank (LTR) and six texture analysis techniques	37 images (sick) and 19 (healthy)	Multi-layer perceptron (MLP) classifier	AUC 98.9%, accuracy 95.8%, recall 97.1%, precision 94.6% (for HOG texture analysis technique)
Sathish and Surekha [19]	Decision tree	Dataset used not specified	Ensemble classifiers (ensemble bagged trees classifier and AdaBoost)	Accuracy 87%, sensitivity 83%, specificity 90.6% (for the ensemble bagged trees classifier)
Torres-Galvan et al. [20]	AlexNet, GoogLeNet, ResNet-50, ResNet-101, inception-v3,VGG-16 and VGG-19	173 images (32 abnormal, 141 healthy)	Pretrained version of network loaded for accuracy, efficient training time	VGG-16 performed best with sensitivity 100%, specificity 82.35%, balanced accuracy 91.18%
Mambou et al. [21]	Deep neural network and SVM (in certain cases)	67 patients (43 healthy, 24 sick)	Pretrained inception V3 model (modification at the last layer)	ROC area 1.00, precision 1.00, recall 1.00
Milosevic et al. [22]	SVM, k-NN, and naive bayes classifier	40 images (26 normal and 14 abnormal)	20 GLCM based texture features are extracted to classify followed by image segmentation	Accuracy 92.5%, sensitivity 78.6% NPV 89.7%
Tello-Mijares et al. [23]	Gradient vector flow with a CNN	63 images (35 normal and 28 abnormal)	Segmentation using GVF followed by CNN	Accuracy 100%, sensitivity 100%, specificity 100%
Hossam et al. [24]	Hough transform (HT) algorithm segmentation	200 images (90 normal and 110 abnormal)	Locate and identify parabolic curves to obtain ROIs	Accuracy 96.667%, kappa statistics 0.9331 (using SVM classifier)
Lou et al. [15]	Segmentation using MultiResUnet neural networks	450 images from 14 patients and 16 volunteers	Segmentation using encoder and a decoder	Average accuracy 91.47% (2 percent higher than an auto encoder)
Roslidar et al. [25]	DenseNet, ResNet101, MobileNetV2, and shuffleNetV2	3581 images (731 cancerous and 2850 healthy)	Tuning the parameters of models to reduce training time while maintaining high accuracy	Best considering train time was MobileNetV2 (static) accuracy 100%, recall 100%, precision 100%
Ahmed et al. [26]	Ant colony optimization and particle swarm optimization	118 frontal views of Patients (30 normal, 45 benign, 43 malignant)	Feature extraction (grey level occurrence matrix) feature selection (ACO and PSO)	ACO: accuracy 94.29%, sensitivity 94.3%, specificity 97.3 PSO: accuracy 97.14%, sensitivity 98%, specificity 98.6%
Nicandro et al. [27]	Bayesian networks	98 cases (77 patients with breast cancer and 21 cases are healthy patients)	Uses hill-climber algo., repeated hill-climber algo. and naive bayes classifier to classify dataset with 14 features	Repeated hill-climber shows best results: accuracy 76.12%, sensitivity 99%

**Table 3:** Machine identification methods.

CNN model	Description
ResNet	Residual networks make use of residual blocks to train very deep neural networks. Making use of these blocks helps prevent the complications that come with training deep networks such as accuracy degradation. The key idea behind these blocks is to have the output of one layer be sent as an input to a layer deeper in the network. This is then added with layer's output in its normal path before the nonlinear function is applied. The variants of ResNet include ResNet-50, ResNet-1202, ResNet-110, ResNet-164, ResNet-101, and ResNet-152 [30].
DenseNet	In the DenseNet architecture, for any layer in the convolutional neural network, the input will be the concatenated result of the output of all the previous layers in the network. By combining information from the previous layers, the computational power can be reduced. Through these connections across all layers, the model is able to retain more information moving across the network improving the overall performance of the network. The variants of DenseNet are DenseNet-B and DenseNet-BC [31].
MobileNet	MobileNet is an architecture that is implemented for mobile devices. They use depth-wise separable convolutions where the filters are added for individual input channels as opposed to the general CNN models. These each channel separate and stack the convoluted outputs together. The different variants include MobileNetV1 and MobileNetV2 [32].
ShuffleNet	They are efficient convolutional neural networks which use filter shuffling to reduce computational complexity. They can reduce the time required to train a model and are used most commonly in smartphones. Shuffling the filters allows more information to pass the network which increases the accuracy of the network with a limited number of resources. The different ShuffleNet models include ShuffleNetV1 and ShuffleNetV2 [33].

**Table 4:** Advantages and disadvantages of various classifiers.

Approach	Advantages	Disadvantages	Ref
Fuzzy rule-based classifier	The logic leading to a prediction is usually transparent	Increasing the partitioning (i.e., number of divisions) makes the classifier computational expensive	[17]
LTR and texture analysis methods	Enable creation of a “compact descriptive representation” of the thermograms	Ranking order can be altered by small perturbations that could go unnoticed by an individual	[18]
Ensemble classifiers	Produce better results if using a single classifier will not give an accurate result	Computationally expensive and the model can become complex	[19]
Alex net, GoogleNet, ResNet-50, ResNet-101, Inception-v3, VGG-16 and VGG-19	Architecture of VGG 16 compared to others outperforms but smaller architecture like GoogleNet is also preferable	VGG-16 is slow to train and the disk space it requires is inefficient (528 MB)	[20]
DNN	Powerful feature extraction and the modification in the final layer helps classify with a better confidence	Overfitting and computationally expensive	[21]
KNN, SVM, Naive Bayes	Lesser data needed to work on compared to NN. SVM works well with outliers. Less complicated to operate.	KNN and SVM take longer to compute. Naive Bayes assumes features are independent	[22]
Gradient vector flow with a CNN	Segmentation to obtain regions of interest	Edge map function constants are determined using knowledge in the topic	[23]
Hough transform (HT) algorithm segmentation	Can distinctly identify breast boundaries	For objects similar to luck, it can give wrong values	[24, 37]
MultiResUnet neural networks	Requires less time and effort than manual segmentation.	Better encoders and decoders exist in for example GoogleNet	[15]
DenseNet, ResNet101, MobileNetV2 and shuffleNetV2	These models has fast training time maintaining high accuracy	Thermal image identification accuracy can be higher	[25]
Ant colony optimization and particle swarm optimization	Feature extraction and selection help eliminate some irrelevant features and increase accuracy	Time of convergence is uncertain for ACO which could be a setback	[26, 38]
Bayesian networks	Features are considered to be dependent on each other. Ability to visually show this relation properly	Requires complex probabilistic function for better metrics. Poor performance for higher number of features	[27, 39]

**Table 5:** CNN models for different views with their outputs.

Model	Output
Frontal model	[P (Hfront), P (Sfront)]
Right 45° model	[P (Hright45), P (Sright45)]
Left 45° model	[P (Hleft45), P (Sleft45)]
Right 90° model	[P (Hright90), P (Sright90)]
Left 90° model	[P (Hleft90), P (Sleft90)]

**Table 6:** The number of samples is based on their class and set.

Classes	Training set (80%)	Test set (20%)
Healthy	126	31
Sick	67	17

**Table 7:** Evaluation metrics.

Metric	Definition	Formula
True positive (TP)	The number of samples which were predicted positive and actually positive	The number of sick patients correctly classified out of the 17 positive samples
False positive (FP)	The number of samples which were predicted positive and actually negative	The number of sick patients that were incorrectly classified out of the 17 positive samples
True negative (TN)	The number of samples which were predicted negative and actually negative	The number of healthy patients correctly classified out of the 31 negative samples
False negative (FN)	The number of samples which were predicted negative and actually positive	The number of healthy patients incorrectly classified out of the 31 negative samples
Accuracy	The proportion of correct classifications	(*TP* +*TN* )/( *TN* +*TP* +*FN* +*FP*)
Sensitivity (recall)	The proportion of the positive class that got correctly classified	(*TP*)/(*TP*+*FN*)
Specificity	The proportion of the negative class that got correctly classified	(*TN*)/(*TN*+*FP*)
Precision	How good a model is at predicting the positive class	(*TP*)/(*TP*+*FP*)

**Table 8:** Model 1 performance evaluation.

Metric	Without CD (%)	With CD (%)
Accuracy	85.4	93.8
Sensitivity	77.8	88.9
Specificity	90.0	96.7
Precision	82.4	94.1
*F*1 score	80.0	91.4
ROC AUC	89.4	98.7
Precision-recall score	84.1	97.7

**Table 9:** Model 2 performance evaluation.

Metric	Without CD (%)	With CD (%)
Accuracy	81.2	89.6
Sensitivity	75.0	87.5
Specificity	84.4	90.6
Precision	70.6	82.4
*F*1 score	72.7	84.8
ROC AUC	80.2	90.0
Precision-recall score	77.1	92.3

**Table 10:** Individual view performance measures.

Model	View	Accuracy	Sensitivity	Specificity
Model 1	Frontal	0.771	0.882	0.710
	Left 90°	0.583	0.412	0.677
	Right 90°	0.723	0.353	0.936

Model 2	Frontal	0.771	0.824	0.742
	Left 90°	0.604	0.530	0.645
	Right 90°	0.708	0.824	0.645

**Table 11:** Comparison of our work with other methods.

Reference paper	Methodology	Accuracy (%)	Sensitivity (%)	Specificity (%)	ROC AUC (%)
[17]	If-then rules	—	74.17	79.02	—
[18]	Learning to rank (LTR) and six texture analysis techniques	95.8	97.1	—	98.8
[19]	Decision tree	87	83	90.6	-
[21]	Deep neural network and SVM	—	100	—	100
[23]	Gradient vector flow with a CNN	100	100	100	—
[24]	Hough transform algorithm segmentation	96.67		—	—
[15]	Segmentation using MulitResUnet neural networks	91.47	—	—	—
[25]	DenseNet, ResNet101, MobileNetV2, and shuffleNetV2	100	100	100	—
[20]	AlexNet, GoogleNet, ResNet-50, ResNet-101, Inception-v3, VGG-16, and VGG-19	91.8	100	82.35	—
[22]	SVM, KNN and Naive Bayes classifier	92.5	78.6	89.7	—
[27]	Bayesian networks	76.12	99	—	—
[26]	Ant colony optimization (ACO) and particle swarm optimization (PSO)	94.29 (for ACO)	94.3 (for ACO)	97.3 (for ACO)	—
Our work	Multiview CNN classification model 1	93.8	88.9	96.7	98.7
Our work	Multi-view CNN classification model 2	89.6	87.5	90.6	90.0

## Data Availability

The data that was used to obtain the findings can be found in the publicly available Visual DMR dataset [43].
